# RhoB Acts as a Tumor Suppressor That Inhibits Malignancy of Clear Cell Renal Cell Carcinoma

This article has been retracted.

**DOI:** 10.1371/journal.pone.0157599

**Published:** 2016-07-06

**Authors:** Weihao Chen, Shaoxi Niu, Xin Ma, Peng Zhang, Yu Gao, Yang Fan, Haigang Pang, Huijie Gong, Donglai Shen, Liangyou Gu, Yu Zhang, Xu Zhang

**Affiliations:** 1 The State Key Laboratory of Kidney Diseases, Department of Urology, Military Postgraduate Medical College, Chinese People's Liberation Army General Hospital, Beijing, People's Republic of China; 2 Department of Urology, General Hospital of the Navy, Beijing, China; Sapporo Medical University, JAPAN

## Abstract

This study aims to investigate the biological role of RhoB in clear cell renal cell carcinoma (ccRCC). The expression of RhoB was examined in specimens of patients and cell lines by Western blot and Immunohistochemistry. The correlation between RhoB expression and clinicopathologic variables was also analyzed. The effects of RhoB on cell proliferation, cell cycle, cell apoptosis, and invasion/migration were detected by over-expression and knockdown of RhoB level in ccRCC cells via plasmids and RNAi. The results showed that RhoB was low-expressed in ccRCC surgical specimens and cell lines compared with adjacent normal renal tissues and normal human renal proximal tubular epithelial cell lines (HKC), and its protein expression level was significantly associated with the tumor pathologic parameter embracing tumor size(*P* = 0.0157), pT stage(*P* = 0.0035), TNM stage(*P* = 0.0024) and Fuhrman tumor grade(*P* = 0.0008). Further, over-expression of RhoB remarkably inhibited the cancer cell proliferation, colony formation and promoted cancer cell apoptosis, and aslo reduced the invasion and migration ability of ccRCC cells. Interestingly, up-regulation of RhoB could induce cell cycle arrest in G2/M phase and led to cell cycle regulators(CyclineB1,CDK1) and pro-apoptotic protein(casp3,casp9) aberrant expression. Moreover, knockdown of RhoB in HKC cells promoted cell proliferation and migration. Taken together, our study indicates that RhoB expression is decreased in ccRCC carcinogenesis and progression. Up-regulation of RhoB significantly inhibits ccRCC cell malignant phenotype. These findings show that RhoB may play a tumor suppressive role in ccRCC cells, raising its potential value in futural therapeutic target for the patients of ccRCC.

## Introduction

Clear cell renal cell carcinoma (ccRCC) originates from proximal tubule cells, and is one of the most common histological subtypes of renal cell carcinomas. ccRCC is the second leading cause of death among all types of urologic cancers[1, 2]. In fact, approximately 25% to 30% of the patients with ccRCC present metastasis at the time of diagnosis, and overall survival is usually very poor in the follow-up period[3]. Unfortunately, ccRCC is resistant to conventional cytotoxic agents, in addition to surgery[4].Although the new targeted therapies have produced dramatic clinical effects for the treatment of metastatic renal-cell carcinoma (RCC), such targeted therapies remain unsatisfactory because some patients are resistant to therapy [5].Thus, further studies are necessary to investigate the tumorigenesis and progression of ccRCC and to explore new therapeutic targets to improve the efficiency of ccRCC treatment.

RhoB is a member of the Rho family of small GTPases, which regulates actin stress fibers, cytoskeletal actin organization and vesicle transport, in cancer cells, RhoB also modulates proliferation, survival, invasion and angiogenic capacity[6]. Furthermore, RhoB may act as a tumor suppressor in growth control and transformation. RhoB is not mutated in various cancers, but its altered expression and activity are possibly critical to cancer progression and therapeutic responses therapeutic responses[7, 8]. Loss of RhoB expression has been reported in head and neck cancer, lung cancer and gastric cancer[9–11]. RhoB gene knockout in mouse increases the frequency of chemically induced neoplastic transformation[12]. Overexpression of RhoB in human tumor cells results in inhibition of signal transduction pathways involved in oncogenesis and tumor survival, as well as apoptosis[13].

Studies have revealed the putative tumor-suppressive effect of RhoB in human tumor, however, to the best of our knowledge, the function of RhoB in ccRCC remains unclear. In the present study, the relative expression levels of RhoB in ccRCC cell lines and patient specimens were investigated by Western blot and immunohistochemistry. The correlation between RhoB expression and clinicopathological parameters of patients with ccRCC was also analyzed. The biological effects of overexpression and low-expression of RhoB on the malignant phenotypes of ccRCC cell A498,786-O and Caki-1 or normal HKC cells were further examined.

## Materials and Methods

### Ethics Statement

All patients authorized the Written Informed Consent. This study was approved by the Protection of Human Subjects Committee, Chinese People’s Liberation Army (PLA) General Hospital.

### Cell culture and reagents

Human renal proximal tubular epithelial cell line HKC and HK2, and the renal cancer cell lines, including A498, 786-O, 769-P and Caki-1, Caki-2 were preserved in our laboratory. The cells were maintained in DMEM or RPMI 1640 medium (Invitrogen, Carlsbad, CA) containing 10% fetal bovine serum (FBS; Invitrogen), 100 units/ml of penicillin and 100 μg/ml streptomycin in a humidified atmosphere of 5% CO_2_ at 37°C.

### Patients and tissue samples

All ccRCC cases diagnosed clinically and histopathologically were obtained from Chinese People’s Liberation Army General Hospital (Beijing, China) in 2011. The study were approved by the Chinese People’s Liberation Army General Hospital’s Protection of Human Subjects Committee and the informed consent was obtained from all patients. After resection was performed, specimens were promptly frozen in liquid nitrogen and stored at -80°C until use. In addition, parts of each sample were fixed in formalin, embedded in paraffin and stored in our laboratory. Inclusion criterion included: Patients who received radical nephrectomy in our hospital, the pathologic diagnosis was ccRCC, both the tumor specimens and renal tissues were available after surgery. Exclusion criterion were as follows:patients receiving chemotherapy or radiotherapy before surgery, with multiple renal tumors or distant metastasis.The following clinicopathologic information was collected for each patient,including age, sex, tumor size, pT status and TNM stage.

### Protein extraction and Western-blot analysis

Whole cell lysate was extracted from each cell line and surgical specimens in RIPA Lysis Buffer (Santa Cruz Biotechnology) according to the manufacturer’s instructions. Protein concentration was measured using BCA Protein Quantitative Kit (Applygen Technologies). Protein(30μg) from each sample was separated in 8% or 12% SDS–PAGE, and transferred to polyvinylidene fluoride membranes (PVDF membranes, Millipore). The PVDF membranes were blocked with 5% low fat milk and then probed with the primary antibody RhoB(1:1000, Proteintech), CyclineB1(1:1000; Immunoway), CDK1(1:1000; Immunoway), cleaved casp9(1:1000, Epitomics), and cleaved casp3(1:1000, Affinity BioReagents). β-actin(1:1000, ZSGB-BIO) was used as a loading control. Secondary anti-mouse or anti-rabbit antibodies were used at 1:3000 dilutions and the reaction was visualized using an enhanced chemiluminescent Kit (Thermo, IL).

### Immunohistochemistry analysis

The paraffin sections (4 μm in thickness) were deparaffinized in xylene solvent and rehydrated through a graded alcohol series. Endogenous peroxidase was suppressed by incubation with 3% hydrogen peroxide for 20 min. For antigen retrieval, the sections were boiled in a pressure cooker containing 10 mM citrate buffer(pH 6.0) for 5 min. The sections were blocked with goat serum in a humid chamber at room temperature for 30 min to reduce non-specific background staining. The sections were further incubated with anti-RhoB antibody at a dilution of 1:100(Rabbit PolyClonal, Proteintech) overnight at 4°C in a moist tray. The sections were also incubated with HRP-conjugated secondary antibody at room temperature for 1h. Afterward, the specimens were washed thrice in PBS, and stained with a liquid DAB substrate kit(ZSGB-BIO, China). Finally, all sections were lightly counterstained with hematoxylin, dehydrated with ethanol, cleaned with xylene and mounted. Aa a negative control, duplicate sections were immunostained without the primary antibody. RhoB expression was scored as 0 (negative), 1 (mild, 0% to 4% positive cells), 2 (moderate, 5% to 49% positive cells) and 3 (strong, ≥50% positive cells)[14].The IHC results were evaluated by two independent pathologists without the knowledge of the patient information.

### Plasmid construction and cell transfection

The human full-length cDNA fragment of RhoB (GenBank accession no. NM_004040) was obtained using general PCR methods. The construct was sub-cloned into the BamHI / EcoRI site of pcDNA3.0-Flag vector containing an ampicillin resistant gene. pcDNA3.0-Flag-RhoB was then used to over-regulate RhoB expression. The small interfering RNA (siRNA) targeting RhoB was designed with sequence Sense: 5’-ACGUCAUUCUCAUGUGCUUTT-3’; Anti-sense: 5’-AAGCACAUGAGAAUGACGUTT, for negative control (Sense: 5’-UUCUCCGAACGUGUCACGUTT-3’; anti-sense: 5’-ACGUGACACGUUCGGAGAATT-3’). These sequences were designed and synthesized by Shanghai Gene-Pharma Co. (Shanghai, China). The plasmid and siRNA were transfected into A498,786-O and Caki-1 cells using lipo2000 (Invitrogen, Carlsbad, CA) according to the manufacturer’s protocol. The expression levels of RhoB were determined by Western blot analysis.

### Cell proliferation assays

In brief, after transfection was performed for 48h, approximately 2000 live cells were seeded in 96-well plates and incubated at 37°C in a 5% CO_2_ incubator for 5d. At the time points of 0, 1, 2, 3, 4, 5,and 6 days, 20μL of MTS solution (Cell Titer96 Aqueous, Promega, Madison, WI) was added to the culture wells. After incubation was conducted for 2 h at 37°C, absorbance was recorded at 490 nm by using a microplate reader.

### Plate colony formation assay

Cells transfected with plasmid and siRNA were seeded at 300 cells per well in six-well plates and incubated at 37°C for two weeks. The cells were fixed with 70% methanol and then stained with crystal violet. The number of positive colonies (more than 50 cells) was counted. All of the experiments were conducted in triplicates.

### Flow cytometry analysis of cell cycle and apoptosis

The transfected cells were harvested when 70% to 80% confluency was reached. For cell cycle analysis, 2× 10^5^ cells were collected, washed with cold PBS twice and fixed with cold 70% ethanol at 4°C overnight. Afterward, the cells were treated with RNase A for 30 min at 37°C, stained with propidium iodide (PI) solution (BD Biosciences, San Jose, CA) for 30 min at 37℃ according to the manufacturer’s protocol and measured by flow cytometry (BD FACS Caton, USA). Cellquest Pro software (BD Biosciences) was used for data acquisition and analysis. For apoptosis analysis, an AnnexinV-FITC apoptosis detection kit (Beyotime Institute of Biotechnology, China) was used according to the manufacturer’s instructions. In brief, 1× 10^6^ cells were obtained and washed twice with PBS. Afterward, the cells were resuspended in FITC-conjugated annexin V binding buffer, incubated with annexinV-FITC/PI in the dark for 10 min and analyzed by flow cytometry using FloMax software.

### Wound-healing assay

Cells were seeded in a six-well cell culture plate and incubated in medium containing 1% FBS. Confluent monolayer cells were scratched with 200-μl pipette tips. The wells were gently washed twice with the medium to remove detached cells. Pictures were obtained at incubation times of 0 h and 24 h, using a phase contrast microscope with a digital camera. The coverage of scraping area was measured on the basis of viable cells migrating from both sides. The experiments were performed in triplicate

### Cell migration and invasion assays

Migration and invasion assays were performed using uncoated and Matrigel-coated Transwell (Corning Costar Corp., Cambridge, MA) membrane filter inserts with pore size of 8 μm according to the manufacturer’s instructions. Approximately 2×10^4^ cells per well were suspended in 200 μL medium with 1% FBS and then seeded into the upper chambers filled with 500 μL medium containing 10% FBS. The cells were incubated at 37°C for 12 h and 24h for migration and invasion respectively. The cells on the upper surfaces of the Transwell chambers were removed by cotton swabs;the cells on the lower surface of the membrane were fixed and stained with crystal violet solution. The number of cells was counted in five randomly selected microscope fields.

### Statistical analysis

The results were represented as the average from triplicate experiments and expressed as mean±SD. Data were analyzed using the SPSS 18 statistical software package (SPSS Inc, Chicago, IL). Student’ *t*-test was conducted to compare the different groups. The association between RhoB staining and clinicopathogic parameters of patients with ccRCC was evaluated by using the chi-square test or the Fisher’s exact test. *P*-value<0.05 was considered statistically significant.

## Results

### RhoB expression is decreased in ccRCC tissues and cell lines

The RhoB protein expression levels were initially analyzed by Wetern blot in seven paired ccRCC surgical specimens and their corresponding adjacent non-tumorous tissues. The results revealed that the RhoB protein expression was remarkably decreased in tumor tissues(Fig 1A). Seven different cell lines, including HKC, human proximal tubular cells (HK-2) and five ccRCC cell lines(A498, Caki-2, 786-O, 769-P and Caki-1),were used to investigate the RhoB expression by Western blot. RhoB protein expression was markedly decreased in ccRCC cell lines compared with the two normal human proximal tubular cell lines (Fig 1B). To further confirm these observations, we performed immunohistochemical analysis in ccRCC tissues and their adjacent non-tumorous tissues. The results showed that RhoB was predominantly located in the cytoplasm of adjacent non-tumorous tissues and the RhoB staining is various in different tumor stages. (Fig 1C).

**Fig 1:** RhoB expression is downregulated in ccRCC tissues and cell lines. (**A**) RhoB protein expression was detected in surgical specimens of ccRCC and their corresponding adjacent non-tumorous tissues by western blot analysis. (**B**) Expression of RhoB in the ccRCC-derived cell lines A498, Caki-2,786-O, 769-P, Caki-1 and human renal proximal tubular cell lines (HKC and HK2) was detecte by western blot. β-action was used as an internal control. (**C**) RhoB protein expression in ccRCC tissues and the matched noncancerous counterpart of the T1 stage ccRCC tissues. (200×c1, 200×c2, the T1 stage of ccRCC tissues and its corresponding noncancerous tissues; 200×c3,the T2 stage of ccRCC tissues; 200×c4, the T3 stage of ccRCC tissues).

### Relationship between RhoB expression and clinical features

The realtionships between RhoB protein expression and clinical features in ccRCC samples (60 cases) using immunohistochemical analysis were listed in Table 1. A total of 38 males and 22 females were included. Our data indicated that RhoB protein expression were significantly associated with tumor size(*P* = 0.0157), pT stage(*P* = 0.0035), TNM stage(*P* = 0.0024) and Fuhrman tumor grade(*P* = 0.0008). However, no significant correlation was observed between RhoB expression and patients’ age and gender.

**Table 1:** The Correlation between RhoB expression and clinicopathological parameters of ccRCC parients.

		RhoB staining		
Variables	Total(n = 60)	0–1	2–3	P-value
Age(years)				0.4211
<55	11	5	6	
≥55	49	16	33	
Gender				0.8662
Male	38	13	25	
Female	22	8	14	
Tumor size				0.0157
≤7cm	38	9	29	
>7cm	22	12	10	
pTstatus				0.0035
pT1-2	47	12	35	
pT3-4	13	9	4	
TMN stage				0.0024
I-II	43	10	33	
III-IV	17	11	6	
Fuhrman stage				0.0008
G1-2	42	9	33	
G3-4	18	12	6	

### RhoB regulates the proliferation of ccRCC cells *In vitro*

Western blot and immunochemical data indicated that RhoB was aberrantly expressed in ccRCC. Therefore, we hypothesized that RhoB might also be involved in ccRCC development or progression. In this study, we employed the MTS assay to evaluate the effects of RhoB on the regulation of ccRCC cell proliferation. The ccRCC cell lines A498 and Caki-1 and the normal renal cell HKC cells were transfected with pcDNA3.0-Flag-RhoB vector or pcDNA3.0-Flag empty vector, and/or siRNAs targeting RhoB or negative control oligo. Over-expression or downregulation efficiency was monitored at the protein level by western blot (Fig 2A–2C). The cell growth curves showed that the overexpression of RhoB significantly inhibited the growth of Caki-1 cells, by contrast, the growth of cells transfected with si-RhoB didn’t differ in terms of proliferation potential (Fig 2D). We further choose relatively high level of endogenous RhoB of A498 and HKC cell lines to examine the cell proliferation ability through downregulteion of RhoB. The growth curves demonstrated that downregulated of RhoB increased A498 and HKC cell growth(Fig 2E and 2F).To confirm the roles of RhoB, we performed plate colony formation assay. The results of colony formation analysis indicated that overexpression of RhoB remarkably reduced the the number of colony forming of Caki-1 cells, conversely, downregulation of RhoB did not modulate focal formation (Fig 2G). The data of the tests of 786-O cells is similar to that of Caki-1 cells, which is put in the S1 Fig. Taken together, these results suggested that RhoB could be a negative regulator of ccRCC cell proliferation.

**Fig 2:** Effects of RhoB on the abilities of cell proliferation of the tumor and normal kidney cell lines. The over-expression or down-expression efficiency was monitored at the protein level in Caki-1(**A**), A498 (**B**) and HKC (C) by western blot. Proliferation curve by MTS assay showing that Caki-1cells (D) transfected with pcDNA3.0-Flag-RhoB grew much more slowly than those transfected with empty vector, whereas cells transfected with si-RhoB and negative control oligo groups made no difference. MTS assay showed knockdown RhoB accelerated the proliferation velocity in A498 (E) and in HKC cells (**F**). (G) Effect of RhoB in colony formation of Caki-1 cells. Results were shown mean±SD *p<0.05. ***p<0.001. Each experiment was performed in triplicate.

### RhoB induces cell cycle arrest in G2/M Phase in ccRCC cells

Cell cycle distribution was determined by flow cytometry with PI staining of 786-O and Caki-1 cell lines to assess whether RhoB induced cell growth inhibition is mediated by alterations in cell cycle progression. Consistent with growth inhibitory effects, the overexpression of RhoB caused a significant increase in cell distribution in the G2/M phase relative to their respective control group (Fig 3A to 3D). However, the groups transfected with negative control or si-RhoB showed no difference in cell cycle phase distribution. To confirm the cell cycle progress results, we investigated the molecular mechanisms of RhoB. The expressions of cell cycle regulators associated with G2/M phase transformation were further investigated in 786-O cells stably transfected with pcDNA3.0-Flag-RhoB or empty vector by Western blot. The protein levels of cyclinB1 and CDK1 were significantly decreased in cells transfected with pc-DNA3.0-Flag-RhoB (Fig 3E and 3F). These results suggested that RhoB modulates cell cycle progression via expression of cell cycle regulators.

**Fig 3:** Influence of RhoB in 786-O cells and Caki-1 cells on cell cycle distribution. 786-O (**A**) and Caki-1(**C**) cells transfected with pcDNA3.0-Flag-RhoB, compared to empty vector showed a higher percentage in G2/M phase. Cells transfected with si-RhoB and negative control group showed no difference in cycling phase distribution. (**B, D**) The data were shown mean±SD of three independent experiments, each performed in triplicate. (**E**) The expression levels of cyclin B1 and CDK1 were significantly decreased in 786-O cells transfected with pcDNA3.0-Flag-RhoB (*p*<0.05). (**F**) Protein relative expression level is shown in mean±SD of triplicate independent experiments with similar numbers.

### RhoB induces cell apoptosis in ccRCC cells

Evasion of apoptosis is a crucial event during malignant transformation,and recent studies have aslo indicated that RhoB is able to induce apoptosis in various cancer cells [15]. Hence, we investigated the effects of RhoB on ccRCC cell apoptosis induction by flow cytometry. Interestingly, the results showed that the percentage of apoptotic cells dramatically increased in 786-O cells transfected with pcDNA3.0-Flag-RhoB compared with cells transfected with the empty vector. Similarly to the influence on cell cycle, groups transfected with si-RhoB or negative control make no difference in apoptosis assays as well(Fig 4A and 4B). Due to the negative results of downregulation of RhoB in 786-O and Caki-1 cells, we also conducted the apoptotic assays in the A498 cells, of which the expression of RhoB is much higher than that of 786-O and caki-1 cells. The outcome is showed in the S2 Fig. To validate cell apoptosis results, we further investigated the apoptotic protein expression. The expression levels of cleaved caspase-3 and caspase-9 were significantly increased in 786-O cells transfected with pc-DNA3.0-Flag-RhoB(Fig 4C). Taken together, these results could explain to some extent why RhoB overexpression could influence the proliferation of ccRCC cells.

**Fig 4:** RhoB induces cell apoptosis in ccRCC cells. (**A**) The percentage of apoptotic cells dramatically increased in 786-O cells transfected with pcDNA3.0-Flag-RhoB compared to empty vector. (**B**) Cells groups transfected with si-RhoB or negative control made no difference in apoptosis rates. ***p<0.001. (**C**) The expression levels of cleaved caspase-3 and caspase-9 were significantly increased in 786-O cells transfected with pcDNA3.0-Flag-RhoB. All experiments were done in triplicates.

### RhoB regulates the migration and invasion of ccRCC cells *In vitro*

To further explore the roles of RhoB in the regulation of cell mobility, we performed migration/invasion assays and wound healing assay in 786-O cells. In transwell migration/invasion assay, our results demonstrated that the overregulation of RhoB protein level significantly decreased the ability of 786-O cells to invade as well as migrate, which is consistent with the wound healing results. The number of 786-O cells that transmigrated to the lower surface of the Transwell membranes was significantly decreased by nearly 4.59-fold (for invasion) and 5-fold (for migration) after cells transfected with pc-DNA3.0-Flag-RhoB compared to those with the empty vector(Fig 5A and 5B). However, the number of invading and migrating cells in the low-expression RhoB group was not significantly different from that of the negative control group(Fig 5A and 5B).

**Fig 5:** Effects of RhoB in invasion and migration of 786-O cells. The invasion (**A**) and migration (**B**) of 786-O cells transfected with pcDNA3.0-Flag-RhoB decreased nearly 4.59-fold (for invasion) and 5-fold (for migration) after transfection with pc-DNA3.0-Flag-RhoB compared with the empty vector. However, the invasion and migration number in the si-RhoB group presented no significant difference compared to the negative control group. (**C**) 786-O cells transfected with pcDNA3.0-Flag-RhoB exhibited an obvious decrease in migration rate compared to cells transfected with empty vector, si-RhoB and negative control groups at 24h point. The data shown were mean±SD, ***p<0.001. Each experiment was performed in triplicate.

To corroborate the results of migration/invasion assays, we performed the wound healing assay. 786-O cells transfected with pc-DNA3.0-Flag-RhoB exhibited a slower wound-healing rate than those transfected with empty vector, si-RhoB and negative control oligo at the same time points(Fig 5C). Considering the low expression level of RhoB in ccRCC cells, we further examined the migration capability in HKC cell after knockdown of RhoB expression level using transwell and wound healing assay. Experiments revealed that that downregulation of RhoB could promoted cell migration ability in HKC cells (S3 Fig). Thus, these results suggested that RhoB can sufficiently inhibit migration and invasion of ccRCC cells *In vitro*.

## Discussion

Rho family GTPases, including RhoA, RhoB, and RhoC, share more than 85% sequence identity. Nevertheless, these GTPases may play distinct physiological and pathophysiological functions in cells, particularly in carcinogenesis[6]. Compared with RhoA and RhoC, RhoB gene is smaller and contains only one exon[16]. Moreover, RhoB is localized in early endosome or other intracellular membranes,wich can be either farnesylated(RhoB-F)or geranylgeranylated(RhoB-GG) modifications, with a specialized function in endocytosis and vesicle trafficking of cytokine receptors, such as epidermal growth factor receptor[17, 18]. RhoB transcript is also characterized by a half-life of only 30 min, and RhoB expression is rapidly induced by a number of stimuli including: UV irradiation, cytokines, growth factors, genotoxic stress, steroid and toxin treatments[19–21].

Although most Rho proteins influence a variety of important processes in malignant transformation, accumulating evidence indicates a tumor suppressive role of RhoB in cancer. RhoA is reprotedly overexpressed in several types of malignancies including breast cancer, hepatocellular carcinoma and colon cancer[22–24]. RhoC protein has been shown to be correlated with tumor metastasis[25]. In contrast, studies on patient biopsies exhibited that RhoB expression levels are dramatically decreased in several tumor types including head and neck, lung and ovary carcinoma, when tumors become more aggressive and invasive[10, 9, 26]. RhoB is not mutated in some cancers, but its altered expression and activity are likely crucial to cancer progression and therapeutic responses[7, 8]. The loss of RhoB expression was strongly associated with higher aggressiveness, worse survival and progression-free survival in non-small cell lung cancer[27]. These observations indicate that Rho protein dysregulation plays an important role in tumor malignant phenotypes.

The suppression of RhoB by many oncogenes are associated with poor prognosis and drug resistance of many cancers, such as the ErbB family of genes, EGF receptor, Ras/PI3K/Akt pathway. However, ectopic expression of RhoB can antagonize the ability of these oncogenes to induce transformation, inhibit cell proliferation, induce apoptosis in response to DNA damaging drugs and abolishe or reduce tumorigenicity in nude mice.[28–30]. Farnesyl transferase inhibitors (FTI) upregulate RhoB levels and this upregulation of RhoB can mediate phenotypic reversion, growth inhibition, cytoskeletal actin reorganization and apoptosis[31]. These data suggested that RhoB may play a protective role to block a crucial step in oncogenesis, Furthermore, oncogenes may have to downregulate RhoB to induce malignant transformation.

Thus far, the role of RhoB in ccRCC has been poorly understood. In our research, we aimed to identify the expression of RhoB in ccRCC clinical specimens and the corresponding effect on tumorigenesis, proliferation, cell cycle, cell apoptosis and migration/invasion ability of ccRCC cells. Our results revealed that the protein expression levels of RhoB were significantly lower in ccRCC tissues and renal cancer cell lines than in the surrounding non-tumorous tissues and normal renal cells. We further analyzed the clinical significance of RhoB expression in patients with ccRCC. Our data showed that RhoB expression was associated with tumor size, Fuhrman grade and tumor grade of ccRCC, suggesting that RhoB expression is correlated with good prognosis markers. This finding is consistent with the idea that RhoB expression is reduced or lost as tumors become more aggressive and high RhoB protein expression is related to enhanced overall survival of patients.

In order to explore the potential roles of RhoB in ccRCC tumorigenesis, the recombinant plasmid expression RhoB (pcDNA3.0-Flag-RhoB) and siRNA targeting RhoB were used to up-regulate and knockdown of RhoB protein level in ccRCC cells. The results of MTS and plate colony formation assays showed that the upregulated RhoB expression significantly inhibited the proliferation and the colony formation of ccRCC cell lines. However, downregulated RhoB expression has no effect in 786-O and Caki-1 cells, it is likely that RhoB is already downregulated in ccRCC cells. Therefore, we further examined the biological effect after knockdown of RhoB in A498 and the normal renal cells HKC. The results showed that downregulted RhoB in A498 and HKC cells colud promote the cancerous phenotypes, such as cell growth and migration abilities. These provided evidence that RhoB may function as a tumor suppressor in ccRCC carcinogenesis.

Altered RhoB expression affects G2/M phase of the cell cycle and the expression of cyclin protein[32]. Mechanistic investigations have indicated that RhoB mediates transcriptional suppression through accumulation of Cyclin B1 in the cytosol at early times after FTI treatment is administered [33]. The RhoB-dependent mechanism of tumor growth inhibition may occur by upregulating the expression of P21, which is a well-characterized CDK inhibitor[34]. In the present study, we found that the restoration of RhoB expression inhibited cell proliferation by blocking the G2/M phase transition in ccRCC cell lines. The decreased expressions of Cyclin B1 and CDK1 were detected in RhoB overexpression cells. These data illustrated that RhoB modulates cell cycle via expression of cell cycle regulators. Cell suicide processes are also possibly play an important role in limiting cancer progression and therapeutic response. RhoB is necessary to induce apoptotic responses of transformed cells to FTI, DNA damaging agents and some anticarcinogens [35, 36, 30]. Our data showed that over-expression of RhoB remarkably induce the apoptosis of ccRCC cells, and increase apoptotic protein(casp3 and casp9) expression.Site-directed mutagenesis studies have defined the crucial requirement of palmitoylated cysteine 192 and prenylated cysteine 193 for tumor suppressive and proapoptotic activities of RhoB [37].

Invasion and migration are two main characteristics of metastatic malignancies, which are critical points in cancer progression and major casues of mortality. Recent data showed that loss of RhoB expression promotes migration and invasion of human bronchial cells by activation of AKT1[38]. Kun jiang et al documented the anti-invasive and antimetastatic activities of RhoB. This result is consistent with that described in other studies, in which RhoB expression is decreased as tumors progress from non-invasive carcinoma stages to highly invasive stages[29]. In this study, wound healing and Transwell assays were conducted to verify the potential effect of RhoB on invasion and migration ability of 786-O cells. The results indicated that invasion and migration of 786-O cells transfected with pcDNA3.0-Flag-RhoB plasmid were decreased compared with those transfected with the empty vector.

In conclusion, our results showed that the decreased expression of RhoB mediated higher malignancy potential in ccRCC. RhoB may play an important role in regulation proliferation, cell cycle progress, cell apoptosis and invasion/migration of ccRCC cells. Thus, RhoB acts as a tumor suppressor in ccRCC pathogenesis. Currently, the mortality of patients with ccRCC is increasing. However, no efficient treatment is available for advanced ccRCC[39, 40]. Therefore, appropriate biomarkers and therapeutic targets of ccRCC should developed. This result suggested that RhoB provideed new insights into the improvement of clinical therapeutic strategies for ccRCC.

## Supporting Information

S1 Fig Over-expression of RhoB inhibits the proliferation of 786-O cells. (**A**)The over-expression or down-expression efficiency was monitored at the protein level in 786-O by western blot. (B) Proliferation curve by MTS assay showing that 786-O cells transfected with pcDNA3.0-Flag-RhoB grew much more slowly than those transfected with empty vector, whereas cells transfected with si-RhoB and negative control oligo groups made no difference. (C) Effect of RhoB in colony formation of 786-O cells. Results were shown mean±SD. *p<0.05. ***p<0.001. Each experiment was performed in triplicate.
(TIF)

S2 Fig RhoB knockdown decreased the cell apoptosis of A498 cells. The percentage of apoptotic cells decreased in cells transfected with Si-RhoB-1 and Si-RhoB-2 compared to control. **p<0.01. All experiments were done in triplicates.
(TIF)

S3 Fig Effects of RhoB on the abilities of cell migration and motility of HKC cells in vitro. (**A**) Representative pictures of the cell migration for the control and siRNA groups in HKC cells. (**B**) RhoB knockdown in siRNA group increased the number of the migration cells compared with the control groups in HKC (P = 0.002). (**C**) Confluent monolayer cells scraped with a plastic 200μl pipette tip. After replacing the cell culture medium, the wound closure was photographed at different time points (0, 24h after scraping). In 100 times microscope, areas of scraping cells were counted. (**D**) Downregulation of RhoB markedly increased the cell viability in HKC cells (P<0.001). Each experiment was performed in triplicate.
(TIF)

## References

[1] LjungbergB, CowanNC, HanburyDC, HoraM, KuczykMA, MerseburgerAS, et al EAU guidelines on renal cell carcinoma: the 2010 update. European Urology. 2010;58(3):398–406. 10.1016/j.eururo.2010.06.032 20633979

[2] JemalA, BrayF, CenterMM, FerlayJ, WardE, FormanD. Global cancer statistics. CA Cancer J Clin. 2011;61(2):69–90. 10.3322/caac.20107 21296855

[3] KarakiewiczPI, BrigantiA, ChunFK, TrinhQD, PerrotteP, FicarraV, et al Multi-institutional validation of a new renal cancer-specific survival nomogram. J Clin Oncol. 2007;25(11):1316–22. 1741685210.1200/JCO.2006.06.1218

[4] HudesG, CarducciM, TomczakP, DutcherJ, FiglinR, KapoorA, et al Temsirolimus, interferon alfa, or both for advanced renal-cell carcinoma. N Engl J Med. 2007;356(22):2271–81. 1753808610.1056/NEJMoa066838

[5] RiniBI, AtkinsMB. Resistance to targeted therapy in renal-cell carcinoma. Lancet Oncol. 2009;10(10):992–1000. 10.1016/S1470-2045(09)70240-2 19796751

[6] PrendergastGC. Actin' up: RhoB in cancer and apoptosis. Nat Rev Cancer. 2001;1(2):162–8. 1190580810.1038/35101096

[7] SatoN, FukuiT, TaniguchiT, YokoyamaT, KondoM, NagasakaT, et al RhoB is frequently downregulated in non-small-cell lung cancer and resides in the 2p24 homozygous deletion region of a lung cancer cell line. Int J Cancer. 2007;120(3):543–51. 1709632710.1002/ijc.22328

[8] FritzG, BrachettiC, BahlmannF, SchmidtM, KainaB. Rho GTPases in human breast tumours: expression and mutation analyses and correlation with clinical parameters. Br J Cancer. 2002;87(6):635–44. 1223777410.1038/sj.bjc.6600510PMC2364248

[9] AdnaneJ, Muro-CachoC, MathewsL, SebtiSM, Munoz-AntoniaT. Suppression of rho B expression in invasive carcinoma from head and neck cancer patients. Clin Cancer Res. 2002;8(7):2225–32. 12114424

[10] MazieresJ, AntoniaT, DasteG, Muro-CachoC, BercheryD, TillementV, et al Loss of RhoB expression in human lung cancer progression. Clin Cancer Res. 2004;10(8):2742–50. 1510267910.1158/1078-0432.ccr-03-0149

[11] ZhouJ, ZhuY, ZhangG, LiuN, SunL, LiuM, et al A distinct role of RhoB in gastric cancer suppression. Int J Cancer. 2011;128(5):1057–68. 10.1002/ijc.25445 20473933

[12] LiuAX, RaneN, LiuJP, PrendergastGC. RhoB is dispensable for mouse development, but it modifies susceptibility to tumor formation as well as cell adhesion and growth factor signaling in transformed cells. Mol Cell Biol. 2001;21(20):6906–12. 1156487410.1128/MCB.21.20.6906-6912.2001PMC99867

[13] ChenZ, SunJ, PradinesA, FavreG, AdnaneJ, SebtiSM. Both farnesylated and geranylgeranylated RhoB inhibit malignant transformation and suppress human tumor growth in nude mice. J Biol Chem. 2000;275(24):17974–8. 1077091910.1074/jbc.C000145200

[14] RenJ, LiW, YanL, JiaoW, TianS, LiD, et al Expression of CIP2A in renal cell carcinomas correlates with tumour invasion, metastasis and patients' survival. Br J Cancer. 2011;105(12):1905–11. 10.1038/bjc.2011.492 22075943PMC3251889

[15] KimBK, KimHM, ChungKS, KimDM, ParkSK, SongA, et al Upregulation of RhoB via c-Jun N-terminal kinase signaling induces apoptosis of the human gastric carcinoma NUGC-3 cells treated with NSC12618. Carcinogenesis. 2011;32(3):254–61. 10.1093/carcin/bgq244 21084431

[16] KarnoubAE, SymonsM, CampbellSL, DerCJ. Molecular basis for Rho GTPase signaling specificity. Breast Cancer Res Treat. 2004;84(1):61–71. 1499915510.1023/B:BREA.0000018427.84929.5c

[17] GampelA, ParkerPJ, MellorH. Regulation of epidermal growth factor receptor traffic by the small GTPase rhoB. Curr Biol. 1999;9(17):955–8. 1050858810.1016/s0960-9822(99)80422-9

[18] Fernandez-BorjaM, JanssenL, VerwoerdD, HordijkP, NeefjesJ. RhoB regulates endosome transport by promoting actin assembly on endosomal membranes through Dia1. J Cell Sci. 2005;118(Pt 12):2661–70. 1594439610.1242/jcs.02384

[19] FritzG, KainaB, AktoriesK. The ras-related small GTP-binding protein RhoB is immediate-early inducible by DNA damaging treatments. J Biol Chem. 1995;270(42):25172–7. 755965210.1074/jbc.270.42.25172

[20] JahnerD, HunterT. The ras-related gene rhoB is an immediate-early gene inducible by v-Fps, epidermal growth factor, and platelet-derived growth factor in rat fibroblasts. Mol Cell Biol. 1991;11(7):3682–90. 171077010.1128/mcb.11.7.3682-3690.1991PMC361128

[21] ChenYX, LiZB, DiaoF, CaoDM, FuCC, LuJ. Up-regulation of RhoB by glucocorticoids and its effects on the cell proliferation and NF-kappaB transcriptional activity. J Steroid Biochem Mol Biol. 2006;101(4–5):179–87. 1704624110.1016/j.jsbmb.2006.06.030

[22] HuT, GuoH, WangW, YuS, HanL, JiangL, et al Loss of p57 expression and RhoA overexpression are associated with poor survival of patients with hepatocellular carcinoma. Oncol Rep. 2013;30(4):1707–14. 10.3892/or.2013.2608 23842948

[23] BellizziA, MangiaA, ChiriattiA, PetroniS, QuarantaM, SchittulliF, et al RhoA protein expression in primary breast cancers and matched lymphocytes is associated with progression of the disease. Int J Mol Med. 2008;22(1):25–31. 18575772

[24] BellovinDI, SimpsonKJ, DanilovT, MaynardE, RimmDL, OettgenP, et al Reciprocal regulation of RhoA and RhoC characterizes the EMT and identifies RhoC as a prognostic marker of colon carcinoma. Oncogene. 2006;25(52):6959–67. 1671513410.1038/sj.onc.1209682

[25] BooneB, Van GeleM, LambertJ, HaspeslaghM, BrochezL. The role of RhoC in growth and metastatic capacity of melanoma. J Cutan Pathol. 2009;36(6):629–36. 10.1111/j.1600-0560.2008.01117.x 19222696

[26] LiuY, SongN, RenK, MengS, XieY, LongQ, et al Expression loss and revivification of RhoB gene in ovary carcinoma carcinogenesis and development. PLoS One. 2013;8(11):e78417 10.1371/journal.pone.0078417 24223801PMC3815309

[27] CalvayracO, PradinesA, Raymond-LetronI, RouquetteI, BousquetE, Lauwers-CancesV, et al RhoB Determines Tumor Aggressiveness in a Murine EGFRL858R-Induced Adenocarcinoma Model and Is a Potential Prognostic Biomarker for Lepidic Lung Cancer. Clin Cancer Res. 2014;20(24):6541–50. 10.1158/1078-0432.CCR-14-0506 25320360

[28] JiangK, DelarueFL, SebtiSM. EGFR, ErbB2 and Ras but not Src suppress RhoB expression while ectopic expression of RhoB antagonizes oncogene-mediated transformation. Oncogene. 2004;23(5):1136–45. 1464741510.1038/sj.onc.1207236

[29] JiangK, SunJ, ChengJ, DjeuJY, WeiS, SebtiS. Akt mediates Ras downregulation of RhoB, a suppressor of transformation, invasion, and metastasis. Mol Cell Biol. 2004;24(12):5565–76. 1516991510.1128/MCB.24.12.5565-5576.2004PMC419878

[30] VishnuP, Colon-OteroG, KennedyGT, MarlowLA, KennedyWP, WuKJ, et al RhoB mediates antitumor synergy of combined ixabepilone and sunitinib in human ovarian serous cancer. Gynecol Oncol. 2012;124(3):589–97. 10.1016/j.ygyno.2011.11.019 22115851PMC3468155

[31] PrendergastGC. Farnesyltransferase inhibitors define a role for RhoB in controlling neoplastic pathophysiology. Histol Histopathol. 2001;16(1):269–75. 1119320210.14670/HH-16.269

[32] ZalcmanG, ClossonV, Linares-CruzG, LereboursF, HonoreN, TavitianA, et al Regulation of Ras-related RhoB protein expression during the cell cycle. Oncogene. 1995;10(10):1935–45. 7539118

[33] KamasaniU, HuangM, DuhadawayJB, ProchownikEV, DonoverPS, PrendergastGC. Cyclin B1 is a critical target of RhoB in the cell suicide program triggered by farnesyl transferase inhibition. Cancer Res. 2004;64(22):8389–96. 1554870910.1158/0008-5472.CAN-04-2437

[34] MarlowLA, ReynoldsLA, ClelandAS, CooperSJ, GumzML, KurakataS, et al Reactivation of suppressed RhoB is a critical step for the inhibition of anaplastic thyroid cancer growth. Cancer Res. 2009;69(4):1536–44. 10.1158/0008-5472.CAN-08-3718 19208833PMC2644344

[35] LiuA, CernigliaGJ, BernhardEJ, PrendergastGC. RhoB is required to mediate apoptosis in neoplastically transformed cells after DNA damage. Proc Natl Acad Sci U S A. 2001;98(11):6192–7. 1135384610.1073/pnas.111137198PMC33444

[36] KamasaniU, LiuAX, PrendergastGC. Genetic response to farnesyltransferase inhibitors: proapoptotic targets of RhoB. Cancer Biol Ther. 2003;2(3):273–80. 12878865

[37] WangDA, SebtiSM. Palmitoylated cysteine 192 is required for RhoB tumor-suppressive and apoptotic activities. Journal of Biological Chemistry. 2005;280(19):19243–9. 1571367710.1074/jbc.M411472200

[38] BousquetE, MazieresJ, PrivatM, RizzatiV, CasanovaA, LedouxA, et al Loss of RhoB expression promotes migration and invasion of human bronchial cells via activation of AKT1. Cancer Res. 2009;69(15):6092–9. 10.1158/0008-5472.CAN-08-4147 19602596

[39] CampbellD, WalkerR, MathewT, CraigJ. Commentary on "Influence of industry on renal guideline development". Clin J Am Soc Nephrol. 2007;2(2):211 1769941310.2215/CJN.00300107

[40] BastienL, CulineS, PauleB, LedbaiS, PatardJJ, de la TailleA. Targeted therapies in metastatic renal cancer in 2009. BJU Int. 2009;103(10):1334–42. 10.1111/j.1464-410X.2009.08454.x 19338565

